RETRACTED

# Circular RNA_0120376 regulates microRNA-148b-3 and centrosomal protein 55 to promote non-small cell lung cancer development

**DOI:** 10.1080/21655979.2022.2052647

**Published:** 2022-05-13

**Authors:** Tiantian Du, Shenni Yi, Yuanyuan Wang, Qiang Zhao, Ping Ma, Wei Jiang

**Affiliations:** a Department of Respiratory and Critical Medicine, Yantai Yuhuangding Hospital, Yantai, China; b Chinese Academy of Sciences, Beijing, China

**Keywords:** Circ_0120376, miR-148b-3p, CEP55, NSCLC

## Abstract

Circular RNAs (circRNAs) are non-coding RNAs with covalent closed-loop structures that are vital in regulating diverse pathological processes. This work is aimed to investigate the role of circ_0120376 in non-small cell lung cancer (NSCLC). Circ_0120376, microRNA (miR)-148b-3p, and centrosomal protein 55 (CEP55) mRNA expression in NSCLC tissues and cells were determined using qRT-PCR. The influences of circ_0120376 and miR-148b-3p on the proliferation of NSCLC cell lines were analyzed by CCK-8 and colony formation assays. Apoptosis was analyzed by flow cytometry. Cell migration and invasion were analyzed using the Transwell experiment. Binding relationships between circ_0120376 and miR-148b-3p and between miR-148b-3p and CEP55 3'UTR were investigated using the dual-luciferase reporter experiment and the RIP experiment. Western blot was conducted to analyze the regulatory effect of circ_0120376 and miR-148b-3p on CEP55 expression. We found that circ_0120376 was markedly overexpressed in NSCLC, and its overexpression was positively associated with increased T stage and lymph node metastasis of the patients. Functional experiments unveiled that circ_0120376 enhanced the proliferation, migration and invasion of NSCLC cells and impeded apoptosis, while knocking down circ_0120376 remarkably suppressed the malignant features of NSCLC cells mentioned above. Circ_0120376 could adsorb miR-148b-3p to reduce miR-148b-3p expression, and circ_0120376 could increase CEP55 expression via adsorbing miR-148b-3p. In summary, circ_0120376 contributes to the malignancy of NSCLC cells through a ceRNA mechanism via regulating miR-148b-3p/CEP55 axis. Circ_0120376 is likely to be a potential diagnostic biomarker and therapeutic target for NSCLC.

## Highlights

- Circ_0120376 is a new circRNA involved in NSCLC progression, which is highly expressed in NSCLC tissues, and promotes the malignancy of cancer cells.
- Circ_0120376 negatively regulates the expression of miR-148b-3p in glioma cells.
- Circ_0120376 can promote the expression of CEP55 in glioma cells via repressing miR-148b-3p.

## 1. Introduction

Lung cancer is the malignancy with the highest morbidity and mortality worldwide [1–3]. Non-small cell lung cancer (NSCLC) takes up about 80% of all lung cancer cases [1–3]. Although great progress has been witnessed, the current therapy of NSCLC remains unsatisfactory [4]. Hence, it is imperative to clarify the molecular mechanism of NSCLC progression to develop innovative treatment strategies for NSCLC.

RETRACTED

Circular RNAs (circRNAs) are derived from the reverse splicing of precursor mRNAs and have a circular covalent structure [5]. CircRNAs do not have free 5’ end or 3’ end, making them more resistant to the degradation induced by RNase or RNA exonucleases [6]. CircRNAs are implicated in the modulation of multiple biological processes in tumor cells, including cell proliferation, differentiation, immune response, apoptosis, migration, and so on [7]. For instance, circ_100395 suppresses lung cancer progression by modulating transcription factor 21 expression [8]. Knocking down circ-ABCB10 can increase the cisplatin sensitivity of lung cancer cells by modulating adenylate kinase 4 expression [9]. It is reported that circ_0120376 (also known as circ-Rtn4) promotes bone marrow-derived mesenchymal stromal cells’ protective function on MC3T3-E1 cells against tumor necrosis factor alpha [10]. Additionally, circ_0120376 exerts a facilitating effect in benzo(a)pyrene-induced transformation of human bronchial epithelial cells [11]. Nonetheless, the role of circ_0120376 in NSCLC is undefined.

MicroRNA (miRNA) is a kind of short RNA transcript of 19 to 25 nucleotides in size that negatively modulates target genes’ expression [12]. MiRNA mimics and miRNA inhibitors have now shown potential as therapeutic agents in the clinic [13]. MiR-148-3p is recognized as a tumor suppressor in several cancers. For example, miR-148b-3p can impede the development of renal cancer cells by modulating fibroblast growth factor-2 [14]. In gastrointestinal stromal tumors, miR-148b-3p directly targets receptor tyrosine kinases KIT to exert tumor-suppressive effects [15]. Nevertheless, the expression pattern and biological function of miR-148b-3p in NSCLC remain unknown.

This work is performed to clarify the role of circ_0120376 in NSCLC. It is hypothesized that circ_0120376 is an oncogenic circRNA in NSCLC, and the current research is performed to validate this. This work reports that circ_0120376 is overexpressed in NSCLC and its overexpression is linked to unfavorable clinicopathological characteristics of NSCLC patients. Functionally and mechanistically, circ_0120376 promotes NSCLC cell proliferation, migration and invasion by moderating the miR-148b-3p/centrosomal protein 55 (CEP55) axis, and impedes apoptosis.

## 2. Materials and methods

### 2.1 Clinical specimens

Cancerous specimens and matched paracancerous tissue specimens were obtained from 113 subjects with newly diagnosed NSCLC at Zhejiang Cancer Hospital. The tissues were acquired during the surgery, and they were preserved in liquid nitrogen until RNA extraction. All tumor tissues and paired paracancerous tissues were confirmed by experienced pathologists after the surgery. The collection and use of human samples was approved by the Ethics Committee of Yantai Yuhuangding Hospital (No. KYC-2018-021).

RETRACTED

### 2.2 Cell culture and transfection

NSCLC cell lines (A549, H596, H2087, and H520) and immortalized lung epithelial cell line 16HBE were procured from the American Type Culture Collection (Manassas, VA, USA). The cells were cultured in Dulbecco’s Modified Eagle Medium (Hyclone, Logan, UT, USA) containing 10% fetal bovine serum, 100 U/mL penicillin, and 100 μg/mL of streptomycin (all from Gibco, Waltham, MA, USA) at 37°C with 5% CO_2_. Circ_0120376 overexpression plasmid pcDNA3.1-circ_0120376 and pcDNA3.1 vector were available from GeneCopoeia (Guangzhou, China). Circ_0120376 specific small interfering RNA (siRNA; si-circ_0120376), miR-148b-3p mimics, miR-148b-3p inhibitors, and corresponding negative controls were designed and synthesized by GenePharma (Shanghai, China). Cell transfection was performed with Lipofectamine^TM^2000 (Invitrogen, Carlsbad, CA, USA) following the protocols.

### 2.3 Quantitative real-time polymerase chain reaction (qRT-PCR)

Total RNA of NSCLC cells or human tissue samples was isolated using TRIzol reagent (Invitrogen, Thermo Fisher Scientific, Inc., Waltham, MA, USA). The RNA concentration was determined by NanoDrop spectrophotometer. RNA was reverse transcribed into cDNA with a reverse transcription kit (Takara, Dalian, China). cDNA was employed as the template, and qRT-PCR was performed on the ABI 7900 Fast RT-PCR System (Applied Biosystems; Thermo Fisher Scientific, Inc., Foster City, CA, USA) with a SYBR Green Master Mix kit (Takara, Otsu, Japan). The primer sequences applied in this experiment are displayed in Table 1.

**Table 1.** Primer sequences used for qRT-PCR

Sequences used for qRT-PCR		
Circ_0120376	Forward	5′-AGTACTTACGAAAGAAGCAGAGG-3′
	Reverse	5′-GTATCACAGGCTCAGATGCAG-3′
CEP55	Forward	5′-AGTAAGTGGGGGATCGAAGCCT-3′
	Reverse	5′-CTCAAGGACTCGAATTTTCTCCA-3′
GAPDH	Forward	5′-CGTGTTCCTACCCCCAATGT-3′
	Reverse	5′-TGTCATCATACTTGGCAGGTTTCT-3′
miR-148b-3p	Forward	5′-TCAGTGCATCACAGAACTTTGT-3′
	Reverse	5′-GCGAGCACAGAATTAATACGAC-3′
U6	Forward	5′-CTCGCTTCGGCAGCACA-3′
	Reverse	5′-AACGCTTCACGAATTTGCGT-3′

### 2.4 Cell counting kit-8 (CCK-8) assay

The cells were inoculated in 96-well plates (2 × 10^3^ cells/well), and the viability of the cells was detected after 24, 48, 72, and 96 h, respectively. At each specific time point, 10 μL of CCK-8 solution (Beyotime, Shanghai, China) was supplemented to each well, and the cells were incubated at 37°C and 5% CO_2_ for 1 h. Then the optical density (D_450 nm_) was measured using a microplate reader.

RETRACTED

### 2.5 Colony formation experiment

Single-cell suspension was added into a 6-well plate (1 × 10^3^ cells/well) and cultured for 14 d. After that, the culture solution was discarded, and the cells were carefully rinsed 3 times with phosphate buffer saline and fixed with 4% paraformaldehyde for 15 min, and stained with 0.5% crystal violet staining solution for 5 min. Ultimately, the colonies were observed and counted with naked eyes.

### 2.6 Flow cytometry

The cells (about 1 × 10^5^ cells) were harvested, cleaned once with phosphate buffer saline, and re-suspended with 500 µL of 1× binding buffer (BioVision, Milpitas, CA, USA). 5 µL of Annexin V-FITC staining solution and 10 µL of PI staining solution (BD Biosciences, San Diego, CA, USA) were supplemented into each sample, and then the cells were incubated in the dark for 30 min. Then the apoptosis was monitored by a flow cytometer (FACScan; BD Biosciences, San Jose, CA, USA).

### 2.7 Transwell experiment

For the migration experiment, 100 μL of cell suspension (the cells were re-suspended in serum-free medium, 1 × 10^5^ cells/mL) was supplemented to the upper compartment of Transwell chamber (Costar, Cambridge, MA, USA), and 500 μL of Dulbecco’s Modified Eagle Medium containing 10% fetal bovine serum was supplemented to the bottom compartment. After 48 h of incubation, the cells attached on the lower surface of the membrane were fixed with paraformaldehyde for 20 min. Subsequently, the fixative solution was discarded, and the cells were stained with 0.5% crystal violet for 20 min. Then cotton swabs were employed to wipe off the cells in the top surface of the membrane. Finally, the stained cells were quantified under a microscope. For the invasion experiment, Matrigel was used to cover the membrane before the cells were inoculated, and the remaining procedures were identical with the migration assay.

### 2.8 Dual-luciferase reporter gene experiment

The binding sites of circ_0120376 and CEP55 3'UTR to miR-148b-3p were screened from by the StarBase database. The circ_0120376-wild type (WT) and circ_0120376-mutant (MUT), CEP55 3'UTR-WT and CEP55 3'UTR-MUT reporter vectors were established based on the psiCHECK-2 vector (Promega, Madison, WI, USA). HEK-293 T cells were co-transfected with miR-148b-3p mimics or negative controls with the reporter vectors, respectively. After 12 h, the luciferase activity of the cells in each group was detected with a dual-luciferase reporter gene assay kit (Beyotime, Shanghai, China) following the protocols.

RETRACTED

### 2.9 RNA immunoprecipitation (RIP)

A Magna RIP^TM^ Kit (Millipore, Billerica, MA, USA) was applied in this assay. Ago2 plasmids or vectors were transfected into NSCLC cell lines, and 1 × 10^7^ cells were collected and suspended in 100 μL of RIP lysis buffer containing protease inhibitor cocktail and RNase inhibitors. The cell lysate was then incubated with 5 μg magnetic bead-coupled anti-Ago2 antibody or anti-IgG antibody overnight at 4°C with rotation. Then RNA molecules were extracted after the protein in the immunoprecipitate was removed by proteinase K. Finally, the abundance of circ_0120376 in the immunoprecipitate was examined by qRT-PCR.

### 2.10 Western blot

NSCLC cells were collected and then the total protein was isolated using radioimmunoprecipitation assay lysis buffer (Beyotime, Shanghai, China). After the sample was mixed with the loading buffer and denatured, the proteins (20 μg/well) were separated by sodium dodecyl sulfate polyacrylamide gel electrophoresis, and then the proteins were transferred onto the polyvinylidene fluoride membrane (Millipore, Billerica, MA, USA). Subsequently, 5% skim milk was employed to block the membrane for 1 h, and then the polyvinylidene fluoride membrane was incubated with anti-CEP55 antibody (Abcam, ab170414, 1:1000) and anti-GAPDH antibody (Abcam, ab9485, 1:1000) overnight at 4°C. The membranes were then rinsed. Subsequently, the secondary antibody (Beyotime, Shanghai, China) was supplemented, and the membrane was incubated for 1 h at room temperature. Ultimately, the membranes were rinsed, and then the protein bands were developed with an ECL substrate kit (Amersham Biosciences, Little Chalfont, UK).

### 2.11 Statistical analysis

All tests were executed for at least three times independently. Statistical analysis was conducted using Statistical Product and Service Solutions (SPSS) (version 18.0) (SPSS, Chicago, IL, USA). Normally distributed data were expressed as mean ± standard deviation. Student’s *t*-test and one-way ANOVA were applied for making the comparison. *p* < 0.05 denoted statistical significance.

## 3. Results

This is a study about the role of circRNA in the tumorigenesis and progression of NSCLC. It is supposed that circ_0120376 is an oncogenic circRNA in NSCLC. In this study, we investigated the expression characteristics, clinical significance, biological function and underlying mechanism of circ_0120376 in NSCLC to verify our hypothesis.

### 3.1 Circ_0120376 was overexpressed in NSCLC and associated with poor clinicopathological parameters

First, circ_0120376 expression in 113 pairs of NSCLC tissues/adjacent tissues was examined by qRT-PCR, and circ_0120376 expression was found to be markedly higher in the cancerous tissues compared with that in the paracancerous tissues (Figure 1A). Additionally, circ_0120376 expression was strongly associated with higher T and N stages of the patients (Figure 1B, C). Moreover, circ_0120376 expression was substantially up-regulated in 4 different NSCLC cell lines when compared with that in 16HBE cell line (Figure 1D). The data implied that circ_0120376 was probably oncogenic in NSCLC.

RETRACTED

**Figure 1.** *Circ_0120376 was overexpressed in NSCLC*. Circ_0120376 expression in human NSCLC tissues and paracancerous tissues was examined by qRT-PCR (n = 113). (b) Circ_0120376 expression was remarkably increased in the cancer tissues of T3 + T4 patients relative to T1+ T2 patients, which was examined by qRT-PCR. (c) qRT-PCR showed that circ_0120376 expression was remarkably increased in the NSCLC tissues of patients with lymph node metastasis. (d) Circ_0120376 expression in 16HBE and 4 types of NSCLC cell lines (A549, H596, H2087, and H520 cells) was detected by qRT-PCR. *P < 0.05, **P < 0.01, ***P < 0.001.

### 3.2 Circ_0120376 enhanced the proliferation, migration and invasion of NSCLC cells, and impeded apoptosis

Next, circ_0120376 overexpression plasmid was transfected into A549 cells to establish the circ_0120376 overexpression model, and si-circ_0120376 was transfected into H520 cells to construct a knockdown model (Figure 2A). CCK-8 experiments and colony formation assays showed that the transfection of circ_0120376 overexpression plasmid markedly facilitated the proliferation of A549 cells (Figure 2B, C). The results of flow cytometry analysis showed a lower rate of apoptosis in A549 cells with circ_0120376 overexpression compared with the cells in the control group (Figure 2D). Additionally, the up-modulation of circ_0120376 remarkably enhanced the migration and invasion of NSCLC cell lines, which was indicated by the Transwell experiments (Figure 2E-F). Conversely, knockdown of circ_0120376 restrained H520 cell proliferation, migration and invasion and facilitated apoptosis (Figure 2B-F).

**Figure 2.** *Circ_0120376 enhanced the proliferation, migration and invasion of NSCLC cells, and restrained apoptosis*. (a) A549 cells were transfected with circ_0120376 overexpression plasmid, and H520 cells were transfected with si-circ_0120376, and successful transfection was proved by qRT-PCR. (b, c) Cell proliferation was monitored using CCK-8 (b) and colony formation (c) assays. (d) Flow cytometry was utilized to examine the apoptosis of NSCLC cells. (e, f) Transwell experiments were adopted to examine NSCLC cell migration (e) and invasion (f). *P < 0.05, ***P < 0.001.

RETRACTED

### 3.3 Circ_0120376 sponged miR-148b-3p

The StarBase database predicted that miR-148b-3p was a candidate target for circ_0120376 (Figure 3A). qRT-PCR revealed that circ_0120376 could negatively modulate miR-148b-3p expression in NSCLC cells (Figure 3B). The analysis of 113 cases of specimens also displayed a remarkably negative correlation between circ_0120376 expression and miR-148b-3p expression (Figure 3C). The data of the dual-luciferase reporter gene assay showed that miR-148b-3p restrained the luciferase activity of wild-type circ_0120376 reporter but had no obvious influence on the luciferase activity of mutated circ_0120376 reporter (Figure 3D). Furthermore, RIP experiments confirmed that circ_0120376 was remarkably enriched with miR-148b-3p in the immunoprecipitate containing Ago2 relative to the IgG group (Figure 3E). Taken together, these findings indicated that circ_0120376 could target miR-148b-3p in NSCLC cells.

**Figure 3.** *MiR-148b-3p was the target of circ_0120376 in NSCLC*. (a) StarBase database predicted a potential binding site between circ_0120376 and miR-148b-3p. (b) qRT-PCR was applied to examine miR-148b-3p expression after up-regulation or knockdown of circ_0120376 in NSCLC cells. (c) Pearson’s correlation analysis showed a negative correlation between miR-148b-3p expression and circ_0120376 expression in NSCLC tissues. (d) Dual-luciferase report assay showed that miR-148b-3p suppressed the luciferase activity of wild type CEP55 reporter, while it had no remarkable effect on the mutant reporter. (e) RIP experiments showed that miR-148b-3 directly interacted with circ_0120376. **P < 0.01, ***P < 0.001.

### 3.4 miR-148b-3p impeded the malignant phenotypes of NSCLC cells

MiR-148b-3p expression was validated to be markedly down-regulated in NSCLC tissues as opposed to the paracancerous tissues using qRT-PCR (Figure 4A). Moreover, miR-148b-3p expression was significantly down-regulated in 4 NSCLC cell lines compared with 16HBE cell line (Figure 4B). To probe the biological function of miR-148b-3p in NSCLC cells, A549 and H520 cells were transfected with miR-148b-3p inhibitors and miR-148b-3p mimics, respectively, and the successful transfection was confirmed by qRT-PCR (Figure 4C). Then, CCK-8 experiment, colony formation assay, Transwell assay and flow cytometry were performed. As shown, inhibiting miR-148b-3p enhanced A549 cell proliferation, migration and invasion and impeded apoptosis, while miR-148b-3p overexpression suppressed the malignant phenotypes of H520 cells (Figure 4D-H). The findings implied that miR-148b-3p was tumor-suppressive in NSCLC.

RETRACTED

**Figure 4.** *miR-148b-3p restrained the proliferation, migration and invasion of NSCLC cells and promoted apoptosis*. (a) MiR-148b-3p expression in NSCLC tissues and paracancerous tissues was analyzed by qRT-PCR. (b) MiR-148b-3p expression in HBE cell line and NSCLC cell lines was analyzed by qRT-PCR. (c) A549 cells were transfected with miR-148b-3p inhibitors, and H520 cells were transfected with miR-148b-3p mimics, and qRT-PCR was utilized to detect the transfection efficacy. (d-h) colony formation assay (d), CCK-8 test (e), Transwell assay (f, g) and flow cytometry (h) were used to detect the effect of miR-148b-3p on the malignant biological behaviors of NSCLC cells. *P < 0.05, **P < 0.01, ***P < 0.001.

### 3.5 miR-148b-3p participated in regulating the malignant phenotypes of NSCLC cells through modulating CEP55

The dataset GSE29249 was analyzed using online GEO2R tool, and the data revealed that CEP55 mRNA was remarkably overexpressed in NSCLC cells (Figure 1A). Consistently, qRT-PCR displayed that CEP55 mRNA was markedly overexpressed in NSCLC tissues and cell lines (Figure 5B, C). Interestingly, StarBase database predicted that, there existed a binding site for miR-148b-3p on the 3'UTR of CEP55 (Figure 5D). As expected, Pearson’s correlation analysis showed a notable negative correlation between miR-148b-3p expression and CEP55 expression in NSCLC specimens (Figure 5E). Additionally, qRT-PCR and Western blot confirmed that miR-148b-3p negatively modulated CEP55 expression at the mRNA and protein levels (figure 5F, G). The data of the dual-luciferase reporter assay manifested that the transfection of miR-148b-3p mimics remarkably restrained the luciferase activity of wild-type CEP55 reporter, whereas it exerted no remarkable effect on mutated CEP55 reporter (Figure 5H). Furthermore, Pearson’s correlation analysis unveiled that circ_0120376 expression was positively correlated with CEP55 mRNA expression in NSCLC specimens (Figure 5I). Furthermore, miR-148b-3p mimic was proved to reverse the promotive effect of circ_0120376 on CEP55 expression, while the miR-148b-3p inhibitors attenuated the suppressing effect of circ_0120376 knockdown on CEP55 expression in NSCLC cells (Figure 5J, K). These data showed that CEP55 was a target gene of miR-148b-3p in NSCLC, and it could be positively modulated by circ_0120376 in NSCLC. Notably, CEP55 knockdown reversed the enhanced proliferation of A549 cells induced by circ_0120376 overexpression, which suggested that circ_0120376 exerted its biological function partly via CEP55 (Supplementary Figure 1).

**Figure 5.** *CEP55 was a direct target of miR-148b-3p in NSCLC cells*. (a) The dataset GSE29249 was analyzed using GEO2R, and the results showed that CEP55 was dysregulated in NSCLC. (b) CEP55 mRNA expression in NSCLC tissues and paracancerous tissues was analyzed by qRT-PCR. (c) CEP55 mRNA expression in NSCLC cell lines was analyzed by qRT-PCR. (d) StarBase database predicted a binding site between miR-148b-3p and CEP55 3'UTR. (e) Pearson’s correlation analysis suggested that miR-148b-3p was negatively correlated with CEP55 expression in NSCLC tissues. (f, g) qRT-PCR (f) and Western blot (g) showed that miR-148b-3p overexpression remarkably inhibited CEP55 expression at the mRNA and protein levels. (h) MiR-148b-3p significantly inhibited the luciferase activity of wild type CEP55 reporter but had no significant effect on that of mutant CEP55 reporter. (i) The Pearson’s correlation analysis suggested that miR-148b-3p expression was positively correlated with circ_0120376 expression in NSCLC tissues. (j, k) qRT-PCR (j) and Western blot (k) were used to detect the expression of CEP55 in NSCLC cells after circ_0120376 and miR-148b-3p were selectively regulated. *P < 0.05, **P < 0.01, ***P < 0.001.

RETRACTED

## 4. Discussion

CircRNA is a class of highly conserved RNA molecules that are widely expressed in human tissues [16,17]. Increasing circRNAs are proved to be aberrantly expressed in human malignancies, and they modulate tumorigenesis and cancer progression [18–21]. For instance, circ_0016760 accelerates NSCLC progression by modulating G antigen 1 and is linked to the adverse prognosis of the patients [22]; circ-PRMT5 overexpression can facilitate enhancer of zeste homolog 2 expressions to promote the proliferation of NSCLC cells [23]; circ_0078767 accelerates cancer development by maintaining Ras association domain family member 1 expression in NSCLC [24]. In the research, circ_0120376 was proved to be remarkably overexpressed in NSCLC tissues and cell lines, and circ_0120376 overexpression was markedly associated with higher clinical stage of NSCLC patients. Furthermore, *in vitro* experiments proved that circ_0120376 facilitated the proliferation, migration and invasion of NSCLC cells. The above data implied that circ_0120376 was cancer-promoting during NSCLC progression.

MiRNAs are small non-coding RNA molecules with 18–22 nucleotides in length that can combine with the 3'UTR of target mRNA to modulate target genes’ expression [25]. Alterations in miRNA expression are therefore associated with the pathogenesis of a lot of human diseases [26–28]. MiR-148b-3p represses gastric cancer cell metastasis by targeting the Dock6/Rac1/cdc42 axis [29]. It also restrains the growth and angiogenesis of cancer cells by targeting fibroblast growth factor receptor 2 in renal cancer [14]. In this work, miR-148b-3p was proved to be markedly under-expressed in NSCLC tissues and cell lines, and we demonstrated that it suppressed NSCLC cell proliferation, migration and invasion, and induced apoptosis, suggesting that miR-148b-3p is a tumor-suppressive miRNA in NSCLC.

RETRACTED

Accumulating studies report that circRNAs can interact with miRNAs via miRNA response element, and this interaction is involved in cancer progression. For example, circ_0074027 enhances the malignant phenotypes of NSCLC cells by targeting miR-185-3p [30]; circ_0001649 impedes NSCLC progression by adsorbing miR-331-3p and miR-338-5p [31]. In the research, bioinformatics analysis identified a potential binding site between miR-148b-3p and circ_0120376, which was then validated by luciferase reporter assay and RIP assay. Also, circ_0120376 was demonstrated to negatively modulate miR-148-3p expression in NSCLC cells, and their expressions were negatively correlated in NSCLC samples. These data suggest that circ_0120376 is a molecular sponge for miR-148b-3p in NSCLC. Interestingly, in the data of TCGA, the expression of miR-148b-3p in both lung adenocarcinoma and lung squamous carcinoma is not significantly changed (v.s. normal tissues) (data not shown). This is inconsistent with our data. This is perhaps due to the heterogeneity of the tissue samples.

CEP55 is an essential modulator of cytoplasmic division, and the knockdown of CEP55 disrupts the proper separation of centrosome and cytoplasm during mitosis [32]. Additionally, CEP55 overexpression is associated with genomic instability, and it is considered to be a cancer-associated protein [33]. CEP55 overexpression is validated to facilitate the malignant phenotypes of cancer cells in diverse tumors, including hepatocellular carcinoma, esophageal squamous cell carcinoma, renal carcinoma, glioma, breast cancer and NSCLC [34–41]. CEP55 can facilitate the growth, migration, and invasion of cancer cells by activating the PI3K/Akt signaling pathway [35–38]. CEP55 overexpression is demonstrated to enhance the NSCLC cell proliferation, and its overexpression is positively linked to adverse NSCLC prognosis [40,41]. In this work, we demonstrated that circ_0120376 could indirectly facilitate CEP55 expression via adsorbing miR-148b-3p. Considering that CEP55 is a crucial regulator of PI3K/Akt signaling, the abnormal expressed circ_0120376 may probably activate this pathway to promote NSCLC progression, which requires further investigation in the future.

## 5. Conclusion

Collectively, this work reveals that circ_0120376 is overexpressed in NSCLC and it promotes the malignancy of NSCLC cells. Meanwhile, this work confirms that circ_0120376 enhances CEP55 expression through sponging miR-148b-3p. The results add to our knowledge of the molecular processes behind NSCLC carcinogenesis and offer a new theoretical foundation for NSCLC treatment. Nevertheless, this work is limited to *in vitro* experiments, and further animal experiments are still needed to validate our findings in the following work.

RETRACTED

## Supplementary Material

Supplemental Material

## Data Availability

The data used to support the findings of this study are available from the corresponding author upon request.
